# Object Detection in Medical Images Based on Hierarchical Transformer and Mask Mechanism

**DOI:** 10.1155/2022/5863782

**Published:** 2022-08-04

**Authors:** Yuntao Shou, Tao Meng, Wei Ai, Canhao Xie, Haiyan Liu, Yina Wang

**Affiliations:** ^1^School of Computer and Information Engineering, Central South University of Forestry and Technology, Changsha 410082, Hunan, China; ^2^College of Information Engineering, Changsha Medical University, Changsha 410219, Hunan, China; ^3^Department of VIP Medical Center, The Third Affiliated Hospital of Sun Yat-Sen University, Sun Yat-Sen University, Guangdong, Guangzhou 510630, China

## Abstract

The object detection task in the medical field is challenging in terms of classification and regression. Due to its crucial applications in computer-aided diagnosis and computer-aided detection techniques, an increasing number of researchers are transferring the object detection techniques to the medical field. However, in existing work on object detection, researchers do not consider the low resolution of medical images, the high amount of noise, and the small size of the objects to be detected. Based on this, this paper proposes a new algorithmic model called the MS Transformer, where a self-supervised learning approach is used to perform a random mask on the input image to reconstruct the input features, learn a richer feature vector, and filter out excessive noise. To focus the model on the small objects that are being detected, the hierarchical transformer model is introduced in this paper, and a sliding window with a local self-attention mechanism is used to give a higher attention score to the small objects to be detected. Finally, a single-stage object detection framework is used to predict the sequence of sets at the location of the bounding box and the class of objects to be detected. On the DeepLesion and BCDD benchmark dataset, the model proposed in this paper achieves better performance improvement on multiple evaluation metric categories.

## 1. Introduction

With the continuous development of deep learning technologies, object detection techniques in the medical field have been widely used in many practical medical diagnostic applications, such as detecting exudates in the retina of diabetic patients [1, 2], early tumor detection, and vascular plaque segmentation. In a traditional medical diagnosis, the presence of lesions in an image is normally identified manually by a physician. This is a time-consuming and labor-intensive task. Meanwhile, since the number of images to be observed every day is large, if doctors continue to perform this task repeatedly, it is easy to cause visual fatigue, which leads to misdiagnosis or missed diagnosis. This is an extremely serious mistake. Therefore, the use of deep learning techniques to enable machines to automatically learn features in images and detect abnormal areas plays an essential role in the field of medical detection [3, 4]. However, since the objects to be detected in medical images are small, making the machine filter out most of the background information and accurately identifying the small lesions in the images is still an important challenge in the field of object detection.

For recent object detection, Girshick et al. [5] used the R–CNN model to obtain several candidate frames, then adopted a CNN to obtain the features of the image, and finally used an SVM to classify the objects. To further improve the accuracy of the model, Ren et al. [6] proposed the Faster R–CNN model, which used RPN to select the candidate frames and only needed to extract the features once to complete the classification and regression of the candidate frames. The Faster R–CNN improves the detection speed of the model.

In the related progress of the latest research, Carion et al. [7] proposed DETR, which used CNN to extract features and then encoded and decoded the obtained features through Transformer to obtain the predicted bounding box. Dosovitskiy et al. [8] proposed the Vision Transformer (ViT), which divided the input image into multiple small patches, performed linear transformation using a linear embedding layer, and finally took the transformed feature vector as the input of the Transformer. Instead of using a conventional CNN architecture for image feature extraction, ViT utilized a self-attention mechanism to extract discriminative features in images. Liu et al. [9] proposed the Swin Transformer based on ViT, which used the window attention mechanism to reduce the model complexity of the self-attention mechanism and can achieve high performance in image recognition and object detection.

Compared with CNN, the ability of Transformer to deal with large-scale datasets is much higher than CNN, and the features extracted by Transformer are correlated with each other, which will provide more semantic information for the model.

For object detection in the medical field, Li et al. [10] improved the stability of retinal lesion detection by combining domain adaptive capabilities and fully convolutional embedding networks. Yan et al. [11] used a 3-dimensional convolutional neural network to extract image features and obtain contextual information, which effectively improved the accuracy of lesion detection using a CT scan. Liao et al. [12] used a region suggestion network (RPN) to process the CT data and extended the RPN network to 3D space, which was effective when extracting a 3D background of CT data. Wang et al. [13] used a deep belief network to extract MRI image features of the brains of patients with Alzheimer's disease. Xie [14] et al. proposed the CoTr model, which fully combined the advantages of CNN and Transformer architectures. CoTr first utilized CNN to extract features in 3D medical images and then used Transformer to model long-range dependencies on the extracted feature maps, which enabled accurate semantic segmentation of 3D medical images. Cao et al. [15] proposed the Swin-Unet model, which used the Swin Transformer as a contextual encoder for medical images and then used a symmetric Transformer decoder to recover the spatial resolution of the feature maps. Swin-Unet had achieved good results on multiorgan and heart image segmentation tasks. Wang et al. [16] proposed the TransBTS model, which exploited the Transformer architecture to extract local 3D contextual history information. TransBTS performed significantly on brain tumor segmentation on 3D MRI scans.

Although better performance results could be obtained using these methods for general object detection applications, they were not applicable for small object detection in medical images. In medical images, the part where the lesion occurs is usually concentrated in a very small area, and the objects to be detected are relatively small in size and belong to small targets. Meanwhile, the clarity of the majority of medical images is relatively low, and there is much noise in the image. Applying general object detection algorithms to aid detection is difficult. It is difficult to apply general algorithms in practice because of the low accuracy of the obtained recognition.

The mask mechanism in the image can filter the raw data to remove excessive noise and obtain the richest semantic information. He et al. [17] used the MAE model to randomly mask the patches of the input image, thus, reconstructing the image pixels and obtaining richer semantic information. Wei et al. [18] proposed MaskFeat, which extracted features using an oriented gradient histogram and utilized the mask mechanism to mask the video sequence, before predicting the masked region, which resulted in better performance improvement. Meanwhile, to improve the recognition accuracy of small objects in medical images, we optimize the transformer proposed by Liu et al. [19] and establish a hierarchical transformer model to detect objects. The hierarchical transformer introduces a self-attention mechanism in the sliding window, and the windows are nonoverlapping with each other. Thus, this algorithm enables the model to learn the differences in the features of the components and, thus, focus on the small objects to be recognized. We believe that combining the mask mechanism with the hierarchical transformer model can be well-applied to the detection of small objects in the medical field.

To address the problem that the current model does not consider the low resolution of images in the medical field, more noise and smaller objects to be detected, this paper introduces the mask mechanism to the self-supervised learning of medical images to reconstruct the medical images and filter out the noise information in the images. First, we segment the medical image into multiple patches (16 × 16) and randomly sample them, and second, we mask the sampled patches, so that they do not participate in feature extraction in the encoding stage. Then, we use Vision Transformer as our encoder and decoder. In the feature encoding stage, we input the unmasked patches into the encoder and map the feature vectors corresponding to the patches into the latent feature space. In the feature decoding stage, we input the feature vector obtained by the encoder and the patches without mask operation into the decoder for decoding operation. Finally, the model achieves the purpose of reconstructing the medical image and filtering out the noise information in the image by continuously narrowing the gap between the input image and the decoded image. In addition, in order to reflect the important difference between different patches in the image in the feature extraction process, we input the feature vector with rich semantic information obtained through the mask self-supervised learning mechanism into the hierarchical Transformer and introduce a nonoverlapping windows self-attention mechanism to learn the important difference between feature vectors. First, we divide the feature vectors of the image into nonoverlapping windows. It used the window attention mechanism to calculate the weight of the feature vectors of each window and gives a higher weight to the window where the small object to be detected is located, so that the model can better adapt to the application scenario of the object detection in small object areas.

The main contributions made in this paper are as follows:

1. In this paper, we propose an algorithm called the MS Transformer for the medical field. By combining the mask mechanism with the hierarchical transformer model, we consider the low resolution of images in the medical field, the high amount of noise, and the small object to be recognized. It can be applied in multimodal image object detection.
2. In this paper, the mask mechanism is successfully applied to the field of target detection, which facilitates image reconstruction and learns more important features and distributions among data on this basis. The mask mechanism can reduce the amount of data needed for model training.
3. This paper optimizes the self-attention mechanism in the Transformer architecture and uses a nonoverlapping window self-attention mechanism. It performs local attention calculation on each image patch by moving the window and gives the small object a higher attention score to be detected. Compared with global attention computation, the model complexity of local attention computation is smaller.
4. On the benchmark dataset, the MS Transformer considerably outperforms existing models in terms of recognition accuracy for multiple categories.

The rest of the paper is organized as follows: in Section 2, we describe in detail the object detection domain and the commonly used methods in the field of medical detection. In Section 3, we present the dataset we use and the data preprocessing process. In Section 4, we introduce the details of the framework of the medical detection model proposed in this paper. In Section 5, we analyze the experimental results. Finally, in Section 6, we draw experimental conclusions and consider the direction of future research.

## 2. Related Work

Object detection tasks have received much attention from researchers in the last few decades. As deep learning methods continue to make substantial breakthroughs, and since object detection tasks in health care are widely used in clinical practice as part of artificial intelligence medicine, researchers have begun to consider applying object detection tasks to health care [10] to improve the efficiency of physicians by using machines to assist them in diagnosing images.

In the existing research on object detection tasks, there are two directions of mainstream research work. One direction is based on a CNN for object detection, and the other is the transformer architecture for encoding and decoding operations on images as a way to achieve object detection.

In the CNN-based modeling approach, Girshick et al. [5] used the R–CNN to extract several candidate frames in the image and then input the obtained features into the CNN for feature extraction. Finally, the SVM classifier was used for classification. This approach was not an end-to-end model framework and was less efficient. Based on the R–CNN, Girshick et al. [6] proposed the Fast R–CNN, which used spatial pyramidal pooling to map the feature vectors of candidate frames into fixed feature vectors and used a fully connected layer for classification. This was an end-to-end modeling framework with some improvement in recognition accuracy, but it had a slower detection speed. To balance the detection speed and the accuracy of the network, Ren et al. [7] proposed the Faster R–CNN. The method used a new method of extracting candidate frames called the RPN. The RPN predicted the probability of a candidate frame at each location in the image. The Faster R–CNN only needed to extract the features once to obtain the candidate frame, which improved the speed of object detection. He et al. [20] used the Mask R–CNN to extract multiscale features. Richer semantic information was obtained, and the detection effect was improved. Tian et al. [21] used multilayer feature maps to extract semantic information. The model was a single-stage object detector. Wieczorek et al. [22] proposed a lightweight CNN, which followed the principle of maximum simplification, can be well deployed on mobile, and has a very high recognition accuracy.

The transformer was proposed by Vaswani et al. [23], and the model architecture did not use the traditional CNN and RNN models, but it consisted of attention mechanisms. The attention mechanism has better results in modeling long-distance dependencies. The transformer was initially achieved with better results in NLP. Considerable progress was also made in the CV field in the last few years.

In the transformer-based modeling approach, Carion et al. [17] used the DETR to input the feature map into a transformer for encoding and decoding operations and output the predicted bounding boxes. This model did not require the preextraction of candidate frames. To improve the convergence speed of the network based on the DETR, Zhu et al. [24] proposed the Deformable DETR, which employed a deformable attention mechanism to make the network focus on only a small portion of the surrounding key points, making the model converge faster. Zhu et al. [25] proposed the TPH-YOLOv5, which was based on YOLOv5, and added a Transformer prediction head to detect the object of different scales to deal with the changing size of objects. Liu et al. [9] proposed the Swin Transformer model, which extracted the semantic features of each part in an image patch in a hierarchical manner by introducing nonoverlapping self-attention windows. Swin Transformer can greatly reduce the number of parameters of the model. However, it suffered from instability during training on large-scale data.

In lesion detection in the medical field, Hu et al. [26] combined CNN and phase-based filters to segment the contours of tumors and achieved superior results. Wang et al. [27] adopted a modified GoogLeNet to slice and dice breast cancer images, which did not consider the location information of the images. Cao et al. [28] used the YOLO model for breast lesion parts for detection and obtained a high recognition accuracy. Dash et al. [29] proposed a joint model of fast-guided and matched filters, which improved the ability to extract vessel features by subsampling the filtered input image. The method achieved very high accuracy on the DRIVE and CHASE_DB1 benchmark datasets. Wozniak et al. [30] proposed a correlation learning mechanism (CLM) deep learning model, which can effectively assist CNN in extracting rich semantic information from CT brain scan images by selecting appropriate filters. CLM had achieved better performance improvements in both speed and accuracy. Chen et al. [31] proposed TransUNet, which combined the advantages of Transformer architecture and U-Net. On the one hand, the Transformer encoder can perform feature extraction of global context from image blocks, and on the other hand, the decoder can upsample the encoded features to achieve feature map resolution recovery. TransUNet is competitive in medical image segmentation tasks.

Since the backbone network is not able to complete the localization of objects, object detection heads are designed to detect the location of objects and categories from the feature map. In the existing work, there are two main ways to design the detection head. One is based on a two-stage object detector, and the other is based on a one-stage detector. A representative work based on two-stage detectors is the R-CNN series [5–7]. In contrast to the two-stage detector, the one-stage detector accomplishes both the regression task of the bounding box and the prediction task of the object class. The one-stage detector has a faster detection speed, but a lower object recognition accuracy [32]. The most representative series of one-stage detectors are the YOLO series [33–36], the SSD [37], and the RetinaNet [27].

Although relevant research on object detection has yielded good results, these schemes have not been widely used in the medical field, and they have major limitations for object detection in the medical field due to the low resolution of the images, a large amount of noise, and the small size of the objects needing to be detected.

This paper proposes the MS Transformer framework model to address the above problems. The model first splits the input image into multiple regular patches (16 × 16) and randomly masks some of the patches. Second, we input the unmasked patches into the encoder for feature mapping to obtain the latent feature vector of the image. Next, we input the obtained latent feature vector together with the feature vector without mask operation to the decoder for self-supervised learning to reconstruct the image, filter out the noise information in the image, and obtain rich semantics Information and data distribution among features. Then, we input the obtained denoised image feature vector into the hierarchical Transformer, use the local attention mechanism in the sliding window to learn the attention weight of each part in the image, and reduce the error of the loss function to make the model endow a higher attention score for the object to be detected. Finally, to make the model's detection efficiency higher, we use the YOLOv5 single-stage object detection head to complete the bounding box regression task and the object recognition classification task.

## 3. Methodology

To address the problems of low resolution, high noise, and small objects to be detected in the medical field, the MS Transformer framework is proposed to filter the background information in images and give higher attention weight to the objects to be detected. The framework consists of a mask self-supervised pretraining model, a hierarchical Transformer model, and a single-target detection head YOLOv5. First, this paper divides the input image into multiple regular patches and performs mask operation on some of the patches. Secondly, we encode the unmasked patches on this basis to obtain the potential distribution of image features. Then, we input the latent feature vector obtained after encoding together with the feature vector without mask operation into the decoder for self-supervised learning to reconstruct the missing pixels. Therefore, the model can learn the semantic features at the pixel level and remove excessive useless information. Then, the obtained image features are embedded into a hierarchical transformer and given attention weights using a sliding window with a local self-attention mechanism. To distinguish between the two, higher attention weights are given to the features of the object needing to be detected and fewer attention weights to the features of the background information. Finally, to improve the detection efficiency of the model for medical images, we input the feature vector with attention weight into the YOLOv5 single-object detection head, and the regression and classification tasks are performed for the bounding box to be predicted, as well as the class of objects with identification for obtaining the sequence of the set of coordinate values of the bounding box and the labeled class of objects to be detected with maximum probability. The specific framework of the MS Transformer model proposed in this paper is shown in Figure 1.

### 3.1. The Image Reconstruction Layer

In this paper, image reconstruction is performed using a self-supervised learning method based on the masking mechanism, which uses an autoencoder to reconstruct the original signal. Similarly to the existing methods, the method in this paper has an encoder that performs an encoding operation on the input features to map them into a high-dimensional vector. It also has a decoder that performs a decoding operation on the high-dimensional vector as a way to reconstruct the input features.

#### 3.1.1. Masking

Similar to ViT [8], first, in this paper, each medical image is segmented into regular patches, and then, we sample them randomly and mask them. A random mask facilitates the elimination of redundancy and enables the model to learn deep-level features.

#### 3.1.2. Encoder

The encoder in this paper adopts the same architecture as ViT [8], and we input the unmasked patches into the encoder for encoding. To reflect the location differences between the different feature vectors, we embed the location vectors corresponding to the feature vectors into their matching patches and then process them through a series of transformer blocks.

#### 3.1.3. Decoder

The input to the encoder is a whole sequence of medical images consisting of unmasked patches and masked tokens. Each masked token in the image is a feature vector that can be learned as a way to predict and reconstruct the missing pixels. Similar to the encoder, we embed the position vector of the entire ensemble sequence into the entire token ensemble sequence to reflect their position information in the image. The reconstructed image feature vectors are then processed by another series of transformer blocks.

The structure of the self-supervised model with the mask mechanism is shown in Figure 2.

### 3.2. Self-Attention Mechanism

To reflect the differences of feature vectors in different regions of the image and give the higher attention score of the objects needing to be detected in the image, we introduce the self-attention mechanism. In medical images, the objects that need to be detected are usually confined to a small region and contain much noise information in the image, and due to the low resolution of the image, it is difficult for the model to learn useful feature information. Therefore, we use the attention mechanism to capture the most useful semantic information in the input feature vector and assign them higher weights.

To distinguish the importance of different feature vectors in medical images, we designed the following self-attention, assuming that the feature map of the input image is *x*. The feature map is linearly mapped to obtain *f*, *g*, *h*, and the vector representation *Z*_*i*_ for each region in the image is obtained as follows:

(1) $$\begin{array}{c} f\left(x\right)={W_{f}}^{*}x,\\ g\left(x\right)={W_{g}}^{*}x,\\ h\left(x\right)={W_{h}}^{*}x,\\ a_{t,i}=\text{softmax}\left(\frac{\exp\left(e_{t,i}\right)}{\sum_{k=1}^{k}\exp\left(e_{t,i}\right)}\right),\\ e_{t,i}=\frac{f{\left(x_{i}\right)}^{T}g\left(x_{j}\right)}{\sqrt{\left|{\text{d}}_{x}\right|}},\\ Z_{i}=W_{v}\left(\sum_{i=1}^{n}a_{t,i}h\left(x_{i}\right)\right), \end{array}$$

where *f*(*x*), *g*(*x*), and *h*(*x*) are the feature vectors of the feature map *x* after linear transformation, *a*_*t*,*i*_ is the similarity score between the *t*-th position and the corresponding *i*-th region, *W*_*v*_ is the same shape as the feature map *x* and the learnable parameter, d_*x*_ is the dimension of the feature map *x*, and *Z*_*i*_ is the final obtained attention weight.

### 3.3. Self-Attention in Local Windows

To make the model focus its attention on the small objects to be detected, we design the windows in a way that the images are uniformly segmented and introduce a self-attention mechanism in the nonoverlapping sliding windows as a way to give a higher attention score to the small objects needing to be detected. In an image of size *hw*, each window is assumed to consist of MM patches, the computational complexity of a global MSA, and the computational complexity of an MSA associated with the window size. The specific calculation formula is defined as follows:

(2) $$\begin{array}{c} \omega \left(\text{MSA}\right)=4hwC^{2}+2{\left(hw\right)}^{2}C,\\ \omega \left(W-\text{MSA}\right)=4hwC^{2}+2M^{2}hwC. \end{array}$$

However, the local window-based attention module does not have the ability to connect other modules across windows, which will greatly limit the modeling capability. To solve the above problem and maintain the computational power of the local window, this paper uses a shift window partitioning method that is divided into two modules and used alternatively in successive hierarchical transformer blocks. The window partitioning strategy of the first module is to partition the 8 × 8 feature map into two windows of size 4 × 4 (*M*=4), and the window partitioning strategy of the second module is based on the first module. The feature map is divided into windows of size [*M*/2, *M*/2].

The continuous hierarchical transformer is calculated as follows:

(3) $$\begin{array}{c} {\hat{Z}}^{l}=W-\text{MSA}\left(LN\left(Z^{l-1}\right)\right)+Z^{l-1},\\ Z^{l}=\text{MLP}\left(LN\left(Z^{l}\right)\right)+{\hat{Z}}^{l},\\ {\hat{Z}}^{l+1}=\text{SW}-\text{MSA}\left(\text{LN}\left(Z^{l}\right)\right)+Z^{l},\\ Z^{l+1}=\text{MLP}\left(\text{LN}\left(Z^{l-1}\right)\right)+{\hat{Z}}^{l+1}, \end{array}$$

where ${\hat{Z}}^{l}$ and *Z*^*l*^ are feature vectors processed by the W-MSA module, the SW-MSA module, and the MLP module. The W-MSA indicates that the window with an attention mechanism uses a conventional division strategy. The SW-MSA indicates that the window with an attention mechanism uses a shift strategy.

### 3.4. YOLOv5 Architecture

The YOLOv5 architecture for single-stage detection consists of three parts: backbone, neck, and prediction. In the backbone, we input the feature vector extracted after processing by the mask self-supervised learning mechanism and the hierarchical Transformer into the Focus architecture and then go through a series of CBL modules, SSP modules, and BottleneckCSP modules. The CBL module comprises a convolutional layer, BatchNorm, and LeakyRELU. The convolutional layer is composed of a convolutional neural network with 32 convolution kernels, a filter size of 3 × 3, and a stride of 2. BottleneckCSP module is composed of Cross Stage Partial Network, which is mainly used to extract rich semantic information in feature vectors. Unlike Convolutional Neural Networks, Bottleneck can reduce gradient information that is repeated during model training. The SSP module consists of spatial pyramid pooling operations, which are mainly used to extract multiscale features. In the neck, the network comprises a series of connection operations, upsampling operations, CBL modules, and BottleneckCSP modules. YOLOv5 also adds an FPN + PAN structure. The FPN layer transfers multiscale semantic information from top to bottom, and the PAN uploads semantic information for localization from bottom to bottom. In the prediction, the model outputs the classification result of the medical image disease and the coordinates of the bounding box.

## 4. Model Training

### 4.1. Image Reconstruction

We will use the mean square error (MSE Loss) to measure the difference between each pixel in the original image and the reconstructed pixel when using the mask self-supervised learning mechanism to filter excessive noise information in medical images. This gap is used to guide the optimization direction of the model parameters. The definition of the MSE Loss function is as follows:

(4) $$\begin{array}{c} {ℒ}_{\text{MSE}}=\frac{1}{N}\sum_{i=1}^{N}{\left(y_{i}-{\hat{y}}_{i}\right)}^{2}, \end{array}$$

where *N* represents the total number of pixels in each medical image, *y*_*i*_ represents the predicted value of the *i*th pixel value in the image, and *y*_*i*_ represents the true value of the *i*th pixel value in the image. In general, the smaller the value of ℒ_MSE_, the smaller the gap between the image pixel value predicted by the model and the real image pixel value, and the stronger the model's ability to reconstruct the image at this time. Based on the MSE Loss function, the learning objective of image data reconstruction is to obtain the smallest loss value among the predicted values of all samples. The objective function is defined as follows:

(5) $$\begin{array}{c} \underset{\theta }{\min}\sum_{i=1}^{N}{ℒ}_{\text{MSE}}\left(\theta \right), \end{array}$$

where *θ* is all the network parameters of the model in the training process. Generally, when the model obtains the smallest loss value, the training effect of the model is the best.

### 4.2. Lesion Attribute Classification

Since the dataset used in this paper is a multiclassification problem, we use a cross-entropy loss function to classify the lesion classes. This loss function is as follows:

(6) $$\begin{array}{c} L_{i}^{k}\left(\theta \right)=\left(y_{i}^{k}\log\left(p_{i}^{k}\right)+\left(1-y_{i}^{k}\right)\left(1-\log\left(p_{i}^{k}\right)\right)\right), \end{array}$$

where *θ* is a parameter that can be learned in the network, *p*_*i*_^*k*^ is the probability of belonging to the *k*-th lesion category, and *y*_*i*_^*k*^ represents the true value of the lesion categories. The smaller the *L*_*i*_^*k*^(*θ*) is, the better the prediction effect of the model is.

To update the network parameters, we defined the following learning objectives:

(7) $$\begin{array}{c} \underset{\theta }{\min}\sum_{i=1}^{N_{2}}\sum_{k=1}^{N_{1}}L_{k=1}^{N1}L_{i}^{k}\left(\theta \right), \end{array}$$

where *N*_1_ and *N*_2_ represent the number of classes of lesions and the number of samples for network training, respectively. Generally, when the value of the cross-entropy loss function of the model is smaller, the classification accuracy of the model for various diseases is higher.

### 4.3. Bounding Box Prediction

To accomplish the regression task of the bounding box in the object detection task, this paper uses the intersection over union (IoU) as our loss function, which is the ratio of the area of the intersection region and the area of the union region between the predicted and real boxes. The formula is defined as follows:

(8) $$\begin{array}{c} \text{IoULoss}=-\text{ln}\frac{\text{Intersection}\left({\text{box}}_{\text{gt}}{\text{,box}}_{\text{pre}}\right)}{\text{Union}\left({\text{box}}_{\text{gt}}{\text{,box}}_{\text{pre}}\right)}, \end{array}$$

where box_gt_ represents the real box, and box_pre_ represents the prediction box. In general, the smaller the IoULoss is, the closer the coordinates of the ground-truth box and the predicted box are.

To update the network parameters, we define the following learning objectives:

(9) $$\begin{array}{c} \underset{\theta }{\min}\sum_{i=1}^{N}\text{IoULoss}\left(\theta \right), \end{array}$$

where *N* represents the number of samples for network training. In general, the smaller the model's IoU Loss value, the more accurate the model's prediction of the bounding box boundaries.

## 5. Experiments

### 5.1. Implementation Details

We implement our model MS Transformer based on the deep learning framework PyTorch 1.8.0 and the programming language *Python* 3.7. All the network training and testing processes are performed in the hardware model RTX3090 GPU. For the medical benchmark datasets used in this paper, we divide them into training, validation, and test sets with ratios of 70%, 15%, and 15% and set the batch size to 32. The weights of all layers in our network are randomly initialized, and Adam [38] is used to optimize the network weights. We set the learning rate to 1e-4. For the model to be fully trained, we set the maximum number of iterations of the network to 500. Meanwhile, to improve the model's generalization ability on the test set, we set the dropout and L2 regularization weights to 0.5 and 0.0005, respectively.

### 5.2. Datasets Used

In this paper, we propose to use DeepLesion [39], the world's largest dataset of CT medical images thus far, which was developed by the NIHCC team and mined and developed from historical medical domain datasets archived in hospitals. This dataset greatly facilitates the development of computer-aided diagnostic techniques and computer-aided detection techniques in the medical field. On 32,120 axial slices, the dataset contains 10,594 CT studies from 4,427 different patients, and it contains 32,735 lesion annotations [11]. Unlike most current datasets, the DeepLesion dataset has a variety of lesion types, including pulmonary nodules, bone lesions, kidney lesions, and lymph node enlargement. They all have a relatively small diameter range, from 0.21 mm to 342.5 mm. The small diameters of the objects to be detected and a large number of categories to be identified make lesion detection for this dataset a challenging task. In this paper, we evaluate the effectiveness of our model based on this dataset. The division of the training, test, and validation sets in this benchmark dataset, as well as the number of categories to be identified and the evaluation metrics, are shown in Table 1.

The BCDD dataset is a benchmark on blood cells containing 4,888 blood cell images. The BCDD dataset has three categories: WBC (white blood cells), RBC (red blood cells), and Platelets, and each image has a label. The dataset shows 4,155 images of the white blood cells category, 372 images of red blood cells, and 361 images of Platelets. The size of each image is 416 × 416. This paper will use the BCDD dataset as another benchmark dataset for our experiments. The division of training set, test set, and validation set in this benchmark dataset, as well as the number of categories to be identified and evaluation indicators, are shown in Table 1.

### 5.3. Baselines and State of the Art

The paper compares the following baseline models with our model:

#### 5.3.1. Fast R–CNN

The Fast R–CNN proposed by Girshick et al. [6] used spatial pyramidal pooling to extract features of candidate frames. The obtained features were then mapped into a fixed-length feature vector. However, this model had limitations and low detection speed, as it used the same method as R–CNN in selecting candidate frames.

#### 5.3.2. Faster R–CNN

The Faster R–CNN proposed by Ren et al. [7] was different from the above methods. It used an RPN network to extract candidate frames, and then the ROI pooling operation was used to unify the size of the feature maps corresponding to the candidate frames. Finally, the classification and the regression tasks were performed on the candidate frames. The model improved the rate of detection, and it was an end-to-end model framework.

#### 5.3.3. Mask R–CNN

To detect objects of different sizes, He et al. [9] proposed Mask R–CNN. The model used an RPN network to extract multiscale features. ROI Align was used to linearly transform the feature map to narrow the gap between the object frame and the candidate frame. The model achieved better results.

#### 5.3.4. DETR

The DETR proposed by Carion et al. [17] treated the object detection task as a prediction task of an ensemble sequence. The DETR used the transformer architecture to encode and decode the input feature map and output the ensemble sequence that predicted the location of the bounding box. The model did not require preextraction of candidate boxes. DETR had a considerable performance improvement.

#### 5.3.5. Swin Transformer

The Swin Transformer proposed by Liu et al. [19] could be used as a backbone network for the object detection task. The model introduced a self-attention mechanism in the sliding window and restricted it to a local window. It enabled the model to assign a larger weight score to the object needing to be detected.

### 5.4. Evaluation Metrics

To verify the effectiveness of the MS Transformer model on the DeepLesion dataset, we use accuracy, *AP*_5_0, and mAP metrics for evaluation.

#### 5.4.1. Accuracy

The accuracy is defined as follows:

(10) $$\begin{array}{c} \text{Accuracy}=\frac{\sum_{j}^{\delta_{1}}A_{j}^{T}}{\sum_{t=1}^{\delta_{2}}x_{i}}, \end{array}$$

where *δ*_1_ and *δ*_2_ are the number of samples in the testing dataset and the correct number of samples predicted by the lesion type, respectively. *x*_*i*_ is the *i*-th lesion sample in the testing dataset, and *A*_*j*_^*T*^ represents the correct prediction of the lesion type of the *j*-th sample. Generally, the larger the accuracy value is, the better the prediction performance of the model is.

#### 5.4.2. AP_5_0

*AP*_5_0 is defined as follows:

(11) $$\begin{array}{c} AP_{5}0=\frac{1}{101}\sum_{0,0.1\ldots 1.0}P_{\text{smooth}}i, \end{array}$$

where 101 represents dividing the range of [0, 1] on the horizontal axis into 100 equal points, and *P*_smooth(*i*)_ represents the precision of the *i*-th point on the smoothed PR curve. *AP*_5_0 represents the IoU threshold of 0.5. In general, the higher the value of *AP*_5_0, the more accurate the coordinate position of the bounding box predicted by the model.

#### 5.4.3. mAP

*mAP* is defined as follows:

(12) $$\begin{array}{c} \text{mAP}=\frac{AP_{50}+AP_{75}+AP_{S}+AP_{M}+AP_{L}}{5}, \end{array}$$

where *AP*_50_ represents the AP value when the IoU threshold is 0.5, *AP*_75_ represents the AP value when the IoU threshold is 0.75, *AP*_*S*_ represents the AP value of the target frame with a pixel area that is less than 32^2^, *AP*_*M*_ represents the AP value of the target frame with a pixel area that is between 32^2^ − 96^2^, and *AP*_*L*_ represents the AP value of the target frame with a pixel area that is greater than 96^2^.

## 6. Results and Discussion

### 6.1. Comparison with the State-of-the-Art and the Baseline

We compare the MS Transformer model proposed in this paper with the current mainstream baseline model and the current state-of-the-art model, DETR. The experimental results show that the model proposed in this paper achieves certain performance improvement in the boundary box prediction task and in the recognition accuracy of lesion categories on the DeepLesion benchmark dataset.

On the DeepLesion dataset, the recognition accuracy of the model in this paper is 90.3%, which is 3.6% higher than that of DETR; the mAP value is 89.6%, which is 1.8% higher than that of DETR. The experimental results demonstrate the effectiveness of our model. The recognition accuracy of lesion types and AP values on bounding box prediction obtained by MS Transformer and other baseline models on the DeepLesion dataset are shown in Tables 2 and 3.

At the same time, we also test the MS Transformer model and other benchmark models on the BCDD benchmark dataset. The experimental results show that MS Transformer has achieved performance improvements in cell location prediction tasks and cell category recognition.

As shown in Tables 4 and 5, on the BCDD dataset, the average recognition accuracy of MS Transformer is 96.15% for cell categories, and it has achieved the best average recognition accuracy. The effect of DETR is second, about 6% lower than that of MS Transformer. The effect of other models is relatively poor, about 12% 21% lower than MS Transformer. MS Transformer achieves the best cell bounding box prediction task results with an mAP value of 91.89%. The effect of Yolov5 is second, which is about 0.2% lower than MS Transformer. The effect of Transformer is slightly worse than that of MS Transformer and Yolov5, with an mAP value of 88.17%. The performance of other models is poor, about 8% 21% lower than MS Transformer.

Compared with the current mainstream baseline models, we believe that the MS Transformer can achieve higher performance on the DeepLesion and BCDD benchmark datasets because of the different application scopes of the model. The model proposed in this paper focuses on object detection tasks in the medical field. Due to the low resolution of medical images and the small objects needing to be detected, we combine the mask mechanism, the hierarchical transformer, and the self-attention mechanism in the images to filter the spurious information and give higher attention weights to the small objects needing to be detected. Although the current state-of-the-art model, DETR, improves on the current mainstream framework Transformer and can achieve substantial results on the Coco dataset, it ignores the image resolution problem. The other baseline models do not consider the image resolution and the size of the objects to be detected. We believe that these two factors will greatly affect the effectiveness of object detection in the medical field.

### 6.2. Ablation Studies

The innovation of our MS Transformer model is the combination of the mask mechanism and the hierarchical transformer model. The mask mechanism is used to reconstruct the input image, and then the hierarchical transformer is used to identify small objects as a solution to the problem of the low resolution of medical images and the small objects needing to be detected. To verify whether the MS Transformer is effective, we conduct ablation experiments on the DeepLesion benchmark dataset, removing one module at a time to check their effects.

The results of the ablation experiments are shown in Table 6. Self-supervised learning through the mask mechanism to reconstruct the input image is beneficial for the model to filter out the spurious information in the image and obtain a feature vector with richer semantic information. If our model does not incorporate the mask mechanism, the accuracy of the model decreases by 8.6%, and the mAP value decreases by 9%. Therefore, we believe that the mask mechanism facilitates the model to better learn the feature distribution among the data.

The experimental results show that the effect of the hierarchical transformer on the model is higher than that of the mask mechanism, and using only the mask mechanism for the object detection task would result in a 15.6% decrease in the accuracy of the model and an 16.1% decrease in the mAP value. We believe that using the local self-attention window in the hierarchical transformer facilitates the model in assigning a greater attention weight to the small objects to be detected, and thus accurately identifying the objects needing to be detected. Therefore, we believe that adding the hierarchical transformer substantially improves the performance of the model.

At the same time, we also conduct ablation experiments with different mask ratios, testing mask ratios ranging from 10% to 80%. As shown in Figure 3, when the mask rate is between 10% and 30%, the recognition accuracy of the model is relatively close, and the accuracy on the BCDD and DeepLesion benchmark datasets is about 86% and 82%, respectively. When the mask rate reaches 40%, the recognition accuracy of the model starts to improve significantly, and the accuracy rates are 94.3% and 87.1%, respectively. Furthermore, on the BCDD benchmark dataset, MS Transformer achieves the highest recognition accuracy when the mask rate is 65%. On the DeepLesion benchmark dataset, MS Transformer achieves the highest recognition accuracy when the mask rate is 75%. Therefore, we believe that the model with mask ratio between 65% and 75% can achieve better results.

## 7. Conclusion

In this paper, we propose an object detection framework in the medical image domain as a way to detect lesion sites. Unlike existing work, the proposed model takes into account the low resolution, high noise, and small objects to be detected in the medical field and provides a richer feature vector for the model. Compared with the existing work, the proposed model achieves higher performance improvement on the DeepLesion benchmark dataset. In future research work, we will consider using RPN networks to extract multiscale features in images as a way to improve the generalization capability of the model. Meanwhile, we also intend to take into account the multimodal features of the images, with the aim of making an important breakthrough at the semantic feature level.

## Figures and Tables

**Figure 1:** The MS Transformer architecture consists of an image reconstruction layer, the Swin Transformer, and the YOLOv5. The hierarchical transformer is composed of two successive transformer blocks. The model finally predicts the lesion class and the bounding box through the fully connected layer and the object detection head, respectively.

**Figure 2:** The image reconstruction layer randomly masks patches of the input image, and then the masked patches are input into the ViT-Transformer for encoding and decoding operations to reconstruct the image by minimizing the loss function.

**Figure 3:** Relationship between mask rate and accuracy on BCDD and DeepLesion benchmark datasets. A high mask rate (65% 75%) can achieve better results.

**Table 1:** Division of the training, test, and validation sets in the DeepLesion dataset and BCDD, as well as the number of categories for detection and the evaluation metrics.

Datasets	Train (%)	Validation (%)	Test (%)	Classes	Evaluation metrics
DeepLesion	70	15	15	8	IoU/mAP/ *AP*_50_
BCDD	70	15	15	3	IoU/mAP/ *AP*_50_

**Table 2:** On the DeepLesion dataset, the MS Transformer compares the recognition accuracy of lesion categories with other baseline models. Acc. = Accuracy.

DeepLesion									
Lesion type	LU	ME	LV	ST	PV	AB	KD	BN	Average (w)
Evaluation metrics	Acc.	Acc.	Acc.	Acc.	Acc.	Acc.	Acc.	Acc.	Acc.
Faster R-CNN	85.9	85.2	88.2	82.0	93.5	81.2	78.4	86.9	83.3
Yolov5	87.2	85.6	86.6	90.9	93.4	84.1	75.5	84.5	85.2
Swin transformer	74.8	84.5	85.6	83.6	93.9	72.9	84.7	83.3	82.9
DETR	89.8	80.7	88.6	94.6	92.7	73.4	77.8	84.4	86.7
MS Transformer	90.7	86.3	94.6	92.9	93.7	71.9	87.9	91.0	90.3

**Table 3:** The *AP*_50_^box^ recognition accuracy of the MS Transformer compared with other baseline models on the DeepLesion dataset.

Methods	DeepLesion								
	LU	ME	LV	ST	PV	AB	KD	BN	Average
	*AP*_50_^box^	*AP*_50_^box^	*AP*_50_^box^	*AP*_50_^box^	*AP*_50_^box^	*AP*_50_^box^	*AP*_50_^box^	*AP*_50_^*box*^	mAP
Faster R-CNN	91.8	81.7	86.5	85.2	89.6	77.0	73.5	81.7	83.3
Yolov5	69.2	90.7	88.1	92.4	95.7	90.6	88.4	90.7	88.2
Swin transformer	21.0	91.5	89.6	92.8	96.4	78.2	88.8	91.1	81.2
DETR	87.9	92.6	90.1	90.5	94.8	90.9	86.2	91.2	87.8
MS Transformer	78.6	89.8	92.3	90.3	97.6	90.2	91.6	92.1	89.6

**Table 4:** On the BCDD dataset, the MS Transformer compares the recognition accuracy of lesion categories with other baseline models. Acc. = Accuracy.

BCDD				
Lesion type	WBC	RBC	Platelets	Average (w)
Evaluation metrics	Acc.	Acc.	Acc.	Acc.
Faster R-CNN	68.71	97.22	63.15	75.46
Yolov5	97.33	77.36	78.21	84.29
Transformer	97.32	79.61	84.53	86.91
DETR	94.25	93.70	84.92	89.86
MS Transformer	100	97.03	94.78	96.15

**Table 5:** The *AP*_50_^box^ recognition accuracy of the MS Transformer compared with other baseline models on the BCDD dataset.

Methods	BCDD			
	WBC	RBC	Platelets	Average
	*AP*_50_^box^	*AP*_50_^box^	*AP*_50_^box^	mAP
Faster R-CNN	35.94	91.70	83.01	70.21
Yolov5	98.21	85.43	91.67	91.67
Transformer	98.84	78.61	87.53	88.17
DETR	76.23	82.35	88.76	83.91
MS Transformer	98.89	90.13	84.31	91.89

**Table 6:** Ablation experiment of the MS Transformer model on the DeepLesion benchmark dataset.

Mask	Hierarchical transformer	Accuracy	mAP
+	−	74.7	73.5
−	+	81.7	80.6
+	+	90.3	89.6

## Data Availability

The dataset used to support the findings of this study are available from the corresponding author upon request.
